# Long non-coding RNA PTPRG-AS1 promotes cell tumorigenicity in epithelial ovarian cancer by decoying microRNA-545-3p and consequently enhancing HDAC4 expression

This article has been retracted.

**DOI:** 10.1186/s13048-020-00723-7

**Published:** 2020-10-24

**Authors:** Juanjuan Shi, Xijian Xu, Dan Zhang, Jiuyan Zhang, Hui Yang, Chang Li, Rui Li, Xuan Wei, Wenqing Luan, Peishu Liu

**Affiliations:** 1 Department of Gynaecology, Qilu Hospital, Cheeloo College of Medicine, Shandong University, 107 West Wenhua Road, Jinan, 277599 Shandong China; 2 Department of Gynaecology, Tengzhou Center People’s Hospital, Zaozhuang, 277500 Shandong China; 3 Department of Gynaecology, Rizhao Central Hospital, Rizhao, 276800 Shandong China; 4 Department of TCM Pharmacy, Tengzhou Center People’s Hospital, Zaozhuang, 277500 Shandong China; 5 Department of Clinical Pharmacy, Tengzhou Center People’s Hospital, Zaozhuang, 277500 Shandong China; 6 Department of Pathology, Tengzhou Center People’s Hospital, Zaozhuang, 277500 Shandong China

**Keywords:** PTPRG antisense RNA 1, Anticancer treatments, Non-coding RNA, ceRNA

## Abstract

**Background:**

Long non-coding RNA PTPRG antisense RNA 1 (PTPRG-AS1) deregulation has been reported in various human malignancies and identified as an important modulator of cancer development. Few reports have focused on the detailed role of PTPRG-AS1 in epithelial ovarian cancer (EOC) and its underlying mechanism. This study aimed to determine the physiological function of PTPRG-AS1 in EOC. A series of experiments were also performed to identify the mechanisms through which PTPRG-AS1 exerts its function in EOC.

**Methods:**

Reverse transcription-quantitative polymerase chain reaction was used to determine PTPRG-AS1 expression in EOC tissues and cell lines. PTPRG-AS1 was silenced in EOC cells and studied with respect to cell proliferation, apoptosis, migration, and invasion in vitro and tumor growth in vivo. The putative miRNAs that target PTPRG-AS1 were predicted using bioinformatics analysis and further confirmed in luciferase reporter and RNA immunoprecipitation assays.

**Results:**

Our data verified the upregulation of PTPRG-AS1 in EOC tissues and cell lines. High PTPRG-AS1 expression was associated with shorter overall survival in patients with EOC. Functionally, EOC cell proliferation, migration, invasion in vitro, and tumor growth in vivo were suppressed by PTPRG-AS1 silencing. In contrast, cell apoptosis was promoted by loss of PTPRG-AS1. Regarding the mechanism, PTPRG-AS1 could serve as a competing endogenous RNA in EOC cells by decoying microRNA-545-3p (miR-545-3p), thereby elevating histone deacetylase 4 (HDAC4) expression. Furthermore, rescue experiments revealed that PTPRG-AS1 knockdown-mediated effects on EOC cells were, in part, counteracted by the inhibition of miR-545-3p or restoration of HDAC4.

**Conclusions:**

PTPRG-AS1 functioned as an oncogenic lncRNA that aggravated the malignancy of EOC through the miR-545-3p/HDAC4 ceRNA network. Thus, targeting the PTPRG-AS1/miR-545-3p/HDAC4 pathway may be a novel strategy for EOC anticancer therapy.

## Background

Ovarian cancer is the seventh most commonly diagnosed human cancer among women [1] and is the most lethal tumor type among gynecologic malignancies [2]. Annually, approximately 220,000 patients are diagnosed with ovarian cancer and 140,000 die of it worldwide [3]. Epithelial ovarian cancer (EOC) is the major pathological type of ovarian cancer and accounts for > 95% of the cases [4]. Roughly 50% of the EOC cases are diagnosed at an advanced stage because of the asymptomatic nature of the disease [5]. Although tremendous progress has been made in diagnostics and therapy over the last decade, treatment remains insufficient and the prognosis remains poor, with a 5-year survival rate of < 30% [6]. The unlimited growth, metastasis, and recurrence are primarily responsible for the poor clinical outcome of EOC patients [7]. In addition, an incomplete understanding of the mechanisms underlying the oncogenesis and progression of EOC has hindered the development of target-based treatment options [8]. Therefore, further studies on the complex etiology and mechanisms implicated in EOC pathogenesis are necessary for identifying the therapeutic targets and improving overall survival.

Long non-coding RNAs (lncRNAs), which comprise approximately 200–10,000 nucleotides, are a heterogeneous group of non-translated RNA transcripts [9]. LncRNAs are widely expressed in a number of tissue types and contribute to cell differentiation, proliferation, metabolism, and other disparate cellular processes [10, 11]. Several studies have revealed lncRNA dysregulation in a wide variety of human cancers and have identified lncRNAs as modulators of tumor etiology and progression [12–14]. Regarding EOC, a substantial amount of evidence has established that various lncRNAs are differentially expressed and function as tumor-inhibiting or tumor-promoting factors in regulating tumorigenesis [15–17].

microRNAs (miRNAs) are a class of single-stranded, non-coding RNA transcripts comprising 17–24 nucleotides [18]. These short miRNAs bind to the 3′-untranslated region (3′-UTRs) of their target genes through miRNA-response elements by complete or incomplete complementary base pairing, which results in translation suppression or target mRNA degradation [19]. miRNAs have also been demonstrated to be crucial regulators of EOC onset and progression and implicated in the control of multiple biological processes [20, 21]. A close correlation between lncRNAs and miRNAs has been demonstrated during carcinogenesis and cancer progression. A competing endogenous RNA (ceRNA) theory asserts that lncRNAs act as specific miRNA sponges and consequently alter the amount of certain mRNAs targeted by miRNAs. Therefore, exploring the function of lncRNAs and miRNAs in EOC as well as elucidating their possible mechanisms of action may provide markers for EOC diagnosis and therapy.

LncRNA PTPRG-AS1 deregulation has been reported to occur in breast cancer [22], nasopharyngeal carcinoma [23], and gastric cancer [24] and was identified as a critical modulator of cancer development. To date, few reports have focused on the detailed role of PTPRG-AS1 in EOC and its underlying mechanisms. This study aimed to elucidate the function of PTPRG-AS1 in EOC. A series of experiments were performed to identify the mechanisms through which PTPRG-AS1 exerts its functions.

## Methods

### Patients and tissue specimens

Fifty-six EOC tissues were collected from patients with EOC in the Qilu Hospital. The clinicopathological characteristics of patients with EOC are shown in Table 1. A total of 21 ovarian surface epithelial tissues were obtained from patients who underwent oophorectomy or hysterectomy for nonmalignant reasons. Patients who had received preoperative radiotherapy or chemotherapy were excluded from the study. All fresh tissues were stored in liquid nitrogen until further use. The study was approved by the Ethics Committee of Qilu Hospital of Shandong University and performed in accordance with the World Medical Association Declaration of Helsinki. Written informed consent was obtained from all participants.

**Table 1:** The clinicopathological characteristics of EOC patients

Clinicopathological characteristics	Case number
**Age (years)**	
< 60	25
≥ 60	31
**Grade**	
G1	26
G2	18
G3	12
**FIGO stage**	
I + II	33
III + IV	23
**Lymphatic metastasis**	
No	24
Yes	32

Abbreviations: *G1* well differentiated, *G2* moderately differentiated, *G3* poorly differentiated, *FIGO* International Federation of Gynecology and Obstetrics

### Cell culture and transfection

Human ovarian surface epithelial (OSE) cells were obtained from ScienCell Research Laboratories (cat. no. 7310) and cultured in ovarian epithelial cell medium (cat. no. 7311; ScienCell Research Laboratories). Four EOC cell lines, ES-2, OVCAR3, CAOV-3, and SK-OV-3, were purchased from the Cell Bank of Type Culture Collection, Chinese Academy of Science (Shanghai, China). McCoy’s 5A (Gibco; Thermo Fisher Scientific, Inc., Waltham, MA, USA) containing 10% fetal bovine serum (FBS; Gibco; Thermo Fisher Scientific, Inc.,) and 1% penicillin/streptomycin (Gibco; Thermo Fisher Scientific, Inc.,) was used to culture ES-2 and SK-OV-3 cells. CAOV-3 cells were cultured in Dulbecco’s modified Eagle’s medium (Gibco; Thermo Fisher Scientific, Inc.,) containing 10% FBS, 1% penicillin/streptomycin mixture, and 1% sodium pyruvate 100 mM solution (Gibco; Thermo Fisher Scientific, Inc.,). RPMI-1640 medium containing 0.01 mg/ml bovine insulin (Gibco; Thermo Fisher Scientific, Inc.,) and 20% FBS was used to the culture OVCAR3 cells. All cells were maintained at 37 °C in a humidified atmosphere with 5% CO_2_.

To silence PTPRG-AS1 expression, EOC cells were transfected with small interfering RNAs (siRNA) targeting PTPRG-AS1 (si-PTPRG-AS1). The negative control siRNA (si-NC) was used as the control for si-PTPRG-AS1. The miR-545-3p mimic, NC mimic, miR-545-3p inhibitor, and NC inhibitor were obtained from Shanghai GenePharma Co., Ltd. (Shanghai, China). The histone deacetylase 4 (HDAC4) overexpressing plasmid pcDNA3.1-HDAC4 (pc-HDAC4) was chemically synthesized by Sangon Biotech Co., Ltd. (Shanghai, China) and used to induce HDAC4 overexpression. EOC cells were collected and seeded into 6-well plates. Cells were grown up to 70–80% confluency and transfected with the molecular products described above using Lipofectamine® 2000 (Invitrogen; Thermo Fisher Scientific, Inc.).

### Reverse transcription-quantitative polymerase chain reaction (RT-qPCR)

RNA was isolated using TRIzol reagent (Invitrogen; Thermo Fisher Scientific, Inc.,). The total RNA was reverse-transcribed to cDNA using the miScript Reverse Transcription Kit (Qiagen GmbH, Hilden, Germany). Quantitative PCR was performed to measure miR-545-3p expression using the miScript SYBR Green PCR Kit (Qiagen GmbH). miR-545-3p expression was normalized to that of U6 small nuclear RNA.

For mRNA detection, reverse transcription was performed with the PrimeScript™ RT reagent Kit (Takara, Dalian, China). PTPRG-AS1 and HDAC4 mRNA expression was quantified by quantitative PCR using the TB Green Premix Ex Taq (Takara). GAPDH was used as an internal control for PTPRG-AS1 and HDAC4. Relative expression was calculated using the 2^−ΔΔCq^ method.

### Cell counting Kit-8 (CCK-8) assay

Transfected cells were collected, counted, and seeded into 96-well plates at a density of 2000 cells per well. After culturing for 0, 24, 48, or 72 h, 10 μl of CCK-8 solution (KeyGen BioTECH; Nanjing, China) was added into each well followed by 2-h incubation at 37 °C in a humidified atmosphere with 5% CO_2_. The absorbance was measured at 450 nm using a microplate reader (BioTek, Winooski, VT, USA).

### Cell apoptosis analysis by flow cytometry

The Annexin V Fluorescein Isothiocyanate (FITC) Apoptosis Detection Kit (Biolegend, San Diego, CA, USA) was used for measuring the relative number of apoptotic cells. Briefly, transfected cells were harvested after 48 h of culture, washed with phosphate buffer saline (PBS), and centrifuged. The collected cells were resuspended in 1× binding buffer and stained with 5 μl annexin V-FITC and 10 μl propidium Iodide. The apoptotic cells were quantified by flow cytometry (FACScan; BD Biosciences, San Jose, CA, USA).

### Transwell cell migration and invasion assays

After 48 h of incubation, transfected cells were trypsinized using 0.25% trypsin, washed with PBS, and resuspended in serum-free culture medium. The concentration of cell suspension was adjusted to 5 × 10^5^ cells/ml. Cell migration assays were performed with the Transwell chambers (8 μM pore size; BD Biosciences), whereas cell invasion assays were performed with the Matrigel-coated chambers (BD Biosciences). The apical chambers were loaded with 200 μL cell suspension, whereas the basolateral chambers were loaded with 500 μl of complete culture medium containing 10% FBS. At 24 h, the cells that had migrated or invaded through the pores were collected with a cotton swab. The migrated and invaded cells were fixed with 5% glutaraldehyde, stained with 0.1% crystal violet, and washed thrice with PBS. After drying, the cells were photographed using an optical microscope (Olympus, Tokyo, Japan). The number of migrated and invaded cells was counted in five randomly selected fields and was considered to be a reflection of the migratory and invasive capacities.

### In vivo tumor xenograft study

The Institutional Animal Care and Use Committee of the Qilu Hospital approved the experiments and procedures involving animals. The in vivo tumor xenograft study was performed in accordance with the National Institutes of Health’s Guide for the Care and Use of Laboratory Animals. The lentivirus plasmids overexpressing PTPRG-AS1 short hairpin RNA (sh-PTPRG-AS1) or NC shRNA (sh-NC) were obtained from Shanghai GenePharma Co., Ltd. and transduced into HEK293T cells in the presence of lentivirus packaging plasmids. The supernatants were collected after 72-h incubation and used to infect CAOV-3 cells. Puromycin (0.5 μg/ml) was used to select CAOV-3 cells stably expressing sh-PTPRG-AS1 or sh-NC. In total, 1 × 10^7^ CAOV-3 cells stably transfected with sh-PTPRG-AS1 or sh-NC were subcutaneously injected into BALB/c nude mice (Beijing Vital River Laboratory Animal Technology Co., Ltd.; Beijing, China). Each group contained three mice. Width and length of tumors were recorded at 4-day intervals for a total of 4 weeks, and the data were used for calculating tumor volumes using the following equation: volume = 0.5 × (length × width^2^). All mice were euthanized, and the tumor xenografts were excised, weighed and analyzed with immunohistochemistry (IHC).

### IHC

HDAC4 and Ki-67expression levels in tumor xenografts were examined via IHC. Tumor xenografts were fixed in 4% neutral formalin and soaked in 4% paraffin, after which the xenografts were cut into 4-μm-thick sections. Deparaffinizing was achieved using xylene, followed by rehydration with an ethanol gradient. Following incubation with 0.3% H2O2 for 30 min and blocking with 5% bovine serum albumin (R&D Systems) for 45 min at 37 °C, the slides were treated with HDAC4 (cat. no. ab235583) or Ki-67 (cat. no. ab15580; all from Abcam) at 4 °C overnight. Thereafter, a horseradish peroxidase-conjugated secondary antibody (cat. no. ab205718; Abcam; 1:500 dilution) was applied to incubate the slides at room temperature for 45 min. Subsequently, 3,3′-diaminobenzidine (DAB) color reagent was added to detect the antibody binding, and tumor xenografts were counterstained with 1% hematoxylin at room temperature for 3 min and dehydrated in ethanol. Image acquisition was conducted using an Olympus microscope.

### Bioinformatics analysis

Two bioinformatics tools, miRDB (http://mirdb.org/) and StarBase 3.0 (http://starbase.sysu.edu.cn/), were used to identify miRNAs that potentially target PTPRG-AS1. The molecular targets of miR-545-3p were predicted using miRDB, StarBase 3.0, and TargetScan (http://www.targetscan.org/).

### Subcellular fractionation

EOC cells were washed with ice-cold PBS and centrifuged. Subcellular fractionation was conducted to isolate cytoplasmic and nuclear fractions of EOC cells using the Nuclear/Cytosol Fractionation Kit (Biovision, San Francisco, CA, USA). The localization of PTPRG-AS1 expression in EOC cells was determined by RT-qPCR analysis.

### Luciferase reporter assay

The wild-type (WT) fragments of PTPRG-AS1 and HDAC4 were amplified and subcloned into the pmirGLO reporter vector (Promega Corporation, Madison, WI, USA). The resulting luciferase reporter plasmids were termed as PTPRG-AS1-WT and HDAC4-WT. Mutation sequences were generated using the Site-Directed Mutagenesis Kit (Agilent, Santa Clara, USA), and the mutant (MUT) fragments were inserted into pmirGLO reporter vectors to obtain PTPRG-AS1-MUT and HDAC4-MUT.

For reporter assays, EOC cells were cotransfected with WT or corresponding MUT reporter plasmids and miR-545-3p mimic or NC mimic using Lipofectamine® 2000. Transfected cells were lysed 48 h after incubation, and the luciferase activity was measured using a Dual-Luciferase Reporter Assay System (Promega Corporation).

### RNA immunoprecipitation (RIP) assay

RIP assay was performed to assess the interaction between miR-545-3p and PTPRG-AS1 in EOC cells following the instructions of Magna RIP RNA-Binding Protein Immunoprecipitation Kit (Millipore, Bedford, MA, USA). A complete RIP lysis buffer was used to lyse the EOC cells, and the cell lysates were incubated at 4 °C with magnetic beads, which were combined with human anti-Argonaute2 (Ago2) antibody or normal mouse IgG (Millipore). After 24 h, the magnetic beads were rinsed and treated with Proteinase K to digest protein. Finally, the immunoprecipitated RNA was analyzed by RT-qPCR to determine the expression of miR-545-3p and PTPRG-AS1.

### Western blotting

RIPA buffer (Beyotime Institute of Biotechnology; Shanghai, China) supplemented with a protease inhibitor cocktail (Beyotime Institute of Biotechnology) was used for total protein extraction. Equal amounts of protein were separated by 10% SDS-PAGE electrophoresis and transferred to PVDF membranes. Tris-buffered saline containing 0.1% Tween-20 (TBST) supplemented with 5% nonfat dried milk was employed for blocking the membranes for 2 h at room temperature. Next, the membranes were incubated with primary antibodies overnight at 4 °C. The primary antibodies against HDAC4 (cat. no. ab235583), E-cadherin (cat. no. ab212059), N-cadherin (cat. no. ab76011), Vimentin (cat. no. ab92547) and GAPDH (cat. no. ab128915) were purchased from Abcam (Cambridge, MA, USA) and used at a dilution of 1:1000. The membranes were washed thrice with TBST and incubated at room temperature for 2 h with a horseradish peroxidase-conjugated secondary antibody (1:5000; cat. no. ab205718; Abcam). Protein bands were visualized using the Immobilon Western Chemilum HRP substrate (Millipore).

### Statistical analysis

All measured data were expressed as the mean ± standard deviation based on at least three independent experiments. Comparisons between two groups were performed with Student’s *t*-test, whereas differences among multiple groups were assessed using one-way ANOVA and Tukey’s post-hoc test. The expression correlation for PTPRG-AS1, miR-545-3p, and HDAC4 was studied using Pearson’s correlation analysis. The overall survival of EOC patients was determined by Kaplan–Meier survival analysis, and the survival curves were compared using the log-rank test. *P* values of < 0.05 were considered statistically significant.

## Results

### Knockdown of PTPRG-AS1 suppresses in vitro EOC cell proliferation, migration, and invasion and promotes cell apoptosis

To elucidate the role of PTPRG-AS1 in EOC, the expression of PTPRG-AS was initially measured in 56 EOC tissues and 21 normal OSE tissues. RT-qPCR analysis confirmed that PTPRG-AS1 expression was elevated in EOC tissues compared with that in normal OSE tissues (Fig. 1a). Similarly, PTPRG-AS1 was highly expressed in four EOC cell lines (ES-2, OVCAR3, CAOV-3, and SK-OV-3) compared with that in human OSE cells (Fig. 1b). The median value for PTPRG-AS1 in EOC was considered the cut-off, and all EOC patients were categorized into PTPRG-AS1-low (*n* = 28) or PTPRG-AS1-high (*n =* 28) groups. Kaplan–Meier survival analysis indicated that patients in the PTPRG-AS1-high group exhibited shorter overall survival than those in the PTPRG-AS1-low group (Fig. 1c; *P* = 0.037).

**Fig. 1:** PTPRG-AS1 silencing inhibits EOC cell proliferation, migration, and invasion but promotes cell apoptosis in vitro. **a** Expression of PTPRG-AS1 in 56 EOC tissues and 21 normal ovarian surface epithelial tissues was measured by RT-qPCR. **b** RT-qPCR measurement of PTPRG-AS1 expression in four EOC cell lines (ES-2, OVCAR3, CAOV-3, and SK-OV-3) and human ovarian surface epithelial (OSE) cells. **c** Overall survival was analyzed in EOC patients according to PTPRG-AS1 expression levels. **d** The knockdown efficiency of si-PTPRG-AS1 was evaluated by RT-qPCR in OVCAR3 and CAOV-3 cells. **e** The proliferation of OVCAR3 and CAOV-3 cells after PTPRG-AS1 depletion was detected by CCK-8 assay. **f** Flow cytometry analysis showed the apoptosis in OVCAR3 and CAOV-3 cells following inhibition of PTPRG-AS1. **g**, **h** The migratory and invasive capacities of OVCAR3 and CAOV-3 cells following PTPRG-AS1 knockdown were determined by Transwell cell migration and invasion assays. **i** The E-cadherin, N-cadherin and Vimentin protein levels in PTPRG-AS1 depleted-OVCAR3 and CAOV-3 cells were examined by western blotting. **P < 0.01

The siRNAs targeting PTPRG-AS1 were transfected into OVCAR3 and CAOV-3 cell lines, and the efficiency of silencing PTPRG-AS1 expression was determined by RT-qPCR. The most efficient siRNA (si-PTPRG-AS1#1) was selected (Fig. 1d), and functional assays were performed to evaluate whether PTPRG-AS1 silencing affects cellular processes in EOC. The CCK-8 assay revealed that the interference of PTPRG-AS1 resulted in an obvious decline in the proliferation of OVCAR3 and CAOV-3 cells (Fig. 1e). Apoptosis of OVCAR3 and CAOV-3 cells increased after PTPRG-AS1 knockdown (Fig. 1f), as demonstrated by flow cytometry. Furthermore, the downregulation of PTPRG-AS1 was linked to a significant decrease in the migration (Fig. 1g) and invasion (Fig. 1h) of OVCAR3 and CAOV-3 cells. Besides, levels of EMT markers, including E-cadherin, N-cadherin and Vimentin, were detected in PTPRG-AS1 depleted-OVCAR3 and CAOV-3 cells. E-cadherin protein level was increased, while N-cadherin and Vimentin levels were reduced in OVCAR3 and CAOV-3 cells after PTPRG-AS1 depletion (Fig. 1i). Collectively, PTPRG-AS1 was upregulated in EOC and exerted oncogenic and malignant effects on EOC cells.

### PTPRG-AS1 “serves as a miR-545-3p” sponge in EOC cells

Substantial studies have indicated that lncRNAs can work as ceRNAs to sequester certain miRNAs in the cytoplasm of cells [25]. The lncLocator (http://www.csbio.sjtu.edu.cn/bioinf/lncLocator/) and lncATLAS (http://lncatlas.crg.eu/) programs were used to predict the localization of PTPRG-AS1. PTPRG-AS1 was predicted to be primarily present in the cytoplasm (Figs. 2a and b). A similar result was obtained by subcellular fractionation using RT-qPCR (Fig. 2c). Bioinformatics tools were used to identify the putative miRNAs that may be sponged by PTPRG-AS1. A total of 14 miRNAs (Fig. 2d) were predicted by both miRDB and StarBase 3.0. Ten miRNAs, including miR-23a-3p [26], miR-23b-3p [27], miR-23c [28], miR-340-5p [29], miR-374c-5p [30], miR-376c-3p [31], miR-383-5p [32], miR-532-5p [33], miR-545-3p [34], and miR-655-3p [35, 36], were selected as candidates for subsequent experiments, considering their implications in cancer oncogenicity.

**Fig. 2:** PTPRG-AS1“serves as a miR-545-3p” sponge in EOC. **a** The distribution of PTPRG-AS1 as predicted by lncLocator. **b** lncATLAS predicts the subcellular localization of PTPRG-AS1. **c** Subcellular fractionation was performed in OVCAR3 and CAOV-3 cells, after which the cytoplasmic and nuclear fractions were analyzed by RT-qPCR for the determination of PTPRG-AS1 subcellular localization. **d** The potential miRNAs that interact with PTPRG-AS1 were predicted by miRDB and StarBase 3.0. **e** The expression of potential target miRNAs in si-PTPRG-AS1-transfected or si-NC-transfected OVCAR3 and CAOV-3 cells was analyzed by RT-qPCR. **f** miR-545-3p expression in 56 EOC tissues and 21 normal ovarian surface epithelial tissues was measured by RT-qPCR. **g** Correlation between the expression of miR-545-3p and PTPRG-AS1 in 56 EOC tissues was analyzed by Pearson’s correlation analysis. **h** The schematic illustration of wild-type and mutant miR-545-3p binding sites within the sequences of PTPRG-AS1. **i** Luciferase reporter assay in OVCAR3 and CAOV-3 cells after cotransfection with miR-545-3p mimic or NC mimic and PTPRG-AS1-WT or PTPRG-AS1-MUT. **j** RIP assay was implemented, and relative enrichment of PTPRG-AS1 and miR-545-3p was detected by RT-qPCR. **P < 0.01

To identify the specific miRNAs contributing to PTPRG-AS1-induced EOC progression, RT-qPCR was performed to determine the expression of the miRNA candidates in OVCAR3 and CAOV-3 cells following PTPRG-AS1 knockdown. The data indicated that the highest expression occurred for miR-545-3p in PTPRG-AS1 deficient-OVCAR3 and CAOV-3 cells, whereas the expression of other miRNAs exhibited no change (Fig. 2e). In addition, miR-545-3p showed reduced expression in EOC tissues compared with that in normal OSE tissues (Fig. 2f). Furthermore, an inverse correlation between miR-545-3p and PTPRG-AS1 was observed in EOC tissues (Fig. 2g; *r* = − 0.6544, *P* < 0.0001).

The luciferase reporter assay was performed to test and verify the specific binding (Fig. 2h) between miR-545-3p and PTPRG-AS1. The upregulation of miR-545-3p resulted in a significant decrease in luciferase activity of PTPRG-AS1-WT; however, luciferase activity was unaffected when the binding sequences were mutated (Fig. 2i). Furthermore, the RIP assay demonstrated that PTPRG-AS1 and miR-545-3p were substantially enriched in the Ago2 antibody-treated group compared with that in the IgG antibody-treated group (Fig. 2j), suggesting that PTPRG-AS1 and miR-545-3p were present in the same RNA-induced silencing complex (RISC). Collectively, these results identified PTPRG-AS1 as a miR-545-3p sponge in EOC.

### miR-545-3p directly targets and regulates HDAC4 in EOC cells

To analyze the role of miR-545-3p in EOC in more detail, miR-545-3p or NC mimic was transfected into OVCAR3 and CAOV-3 cells. Consequently, the expression of miR-545-3p was dramatically increased in miR-545-3p mimic-transfected cells (Fig. 3a). CCK-8 assay revealed that the proliferative ability of OVCAR3 and CAOV-3 cells was reduced after miR-545-3p overexpression (Fig. 3b). In addition, ectopic miR-545-3p expression induced apoptosis in OVCAR3 and CAOV-3 cells (Fig. 3c). Furthermore, overexpressed miR-545-3p clearly impaired the migratory (Fig. 3d) and invasive (Fig. 3e) properties of OVCAR3 and CAOV-3 cells.

**Fig. 3:** HDAC4 is a direct target of miR-545-3p in EOC. **a** The overexpression efficiency of miR-545-3p mimic in OVCAR3 and CAOV-3 cells was examined by RT-qPCR. **b**, **c** CCK-8 assay and flow cytometry analyses were performed to measure the proliferation and apoptosis of OVCAR3 and CAOV-3 cells after miR-545-3p overexpression. **d**, **e** Transwell cell migration and invasion assays assessed the migration and invasion of OVCAR3 and CAOV-3 cells that were transfected with miR-545-3p mimic or NC mimic. **f** The wild-type and mutant putative binding sequences of miR-545-3p in the sequence of the HDAC4 3′-UTR. **g**, **h** The expression levels of HDAC4 mRNA and protein in OVCAR3 and CAOV-3 cells with miR-545-3p upregulation were measured by RT-qPCR and western blot analysis. **i** HDAC4 mRNA expression was measured by RT-qPCR in 56 EOC tissues and 21 normal ovarian surface epithelial tissues. **j** The relationship between HDAC4 mRNA and miR-545-3p in 56 EOC tissues was determined by Pearson’s correlation analysis. **k** miR-545-3p mimic or NC mimic was cotransfected with HDAC4-WT or HDAC4-MUT into OVCAR3 and CAOV-3 cells. The luciferase activity was detected at 48 h post-transfection. **P < 0.01

After revealing the function of miR-545-3p in EOC, mechanistic studies were conducted to identify the targets of miR-545-3p. HDAC4 (Fig. 3f) was predicted as a potential target of miR-545-3p and selected for further verification because of its tumor-promoting role during EOC progression [37–39]. RT-qPCR and western blot analysis revealed that overexpressed miR-545-3p decreased the mRNA (Fig. 3g) and protein (Fig. 3h) expression of HDAC4 in OVCAR3 and CAOV-3 cells. Moreover, HDAC4 was highly expressed in EOC tissues (Fig. 3i) and inversely correlated with miR-545-3p expression (Fig. 3j; *r* = − 0.7369, *P* < 0.0001). Next, luciferase reporter assay was used to validate the binding site between miR-545-3p and the 3′-UTR of HDAC4. The results revealed that cotransfection of miR-545-3p mimic with HDAC4-WT resulted in reduced luciferase activity, whereas miR-545-3p mimic and HDAC4-MUT cotransfection did not alter luciferase activity (Fig. 3k). Collectively, these experiments validated HDAC4 as a direct target of miR-545-3p in EOC cells.

### PTPRG-AS1 promotes the expression of HDAC4 in EOC cells by sponging miR-545-3p

A series of experiments were performed to determine the association among PTPRG-AS1, miR-545-3p, and HDAC4 in EOC. First, RIP assay was performed, and the results showed that PTPRG-AS1, miR-545-3p, and HDAC4 were all enriched in the Ago2 antibody-treated group (Fig. 4a), suggesting that all three molecules co-exist in RISC. Next, RT-qPCR and western blot analysis were conducted to elucidate the regulatory role of PTPRG-AS1 in HDAC4 expression in EOC cells. The loss of PTPRG-AS1 reduced HDAC4 expression at both the mRNA (Fig. 4b) and protein (Fig. 4c) levels in OVCAR3 and CAOV-3 cells, and the inhibitory effects were abolished by synergistically silencing miR-545-3p expression (Figs. 4d and e). In addition, Pearson’s correlation analysis identified a positive correlation between PTPRG-AS1 and HDAC4 mRNA in EOC tissues (Fig. 4f; *r* = 0.7207, *P <* 0.0001). Thus, PTPRG-AS1 functioned as a miR-545-3p sponge to upregulate HDAC4 expression in EOC cells.

**Fig. 4:** PTPRG-AS1 sequesters miR-545-3p and thereby increases HDAC4 expression in EOC. **a** A RIP assay was performed to elucidate whether PTPRG-AS1, miR-545-3p, and HDAC4 exist in the same RISC. **b**, **c** RT-qPCR and western blot analysis were conducted to measure HDAC4 mRNA and protein expression in PTPRG-AS1 deficient OVCAR3 and CAOV-3 cells. **d**, **e** si-PTPRG-AS1 combined with miR-545-3p inhibitor or NC inhibitor were cotransfected into OVCAR3 and CAOV-3 cells, and the expression changes of HDAC4 mRNA and protein were assessed. **f** Pearson’s correlation analysis was applied to examine the relationship between PTPRG-AS1 and HDAC4 mRNA expression in 56 EOC tissues. **P < 0.01

### PTPRG-AS1 depleted-induced cancer-inhibiting actions in EOC cells are implemented by regulating miR-545-3p/HDAC4

To determine whether PTPRG-AS1 functions in EOC by targeting miR-545-3p/HDAC4, miR-545-3p inhibitor or NC inhibitor together with si-PTPRG-AS1 was introduced into EOC cells. The transfection efficiency of miR-545-3p inhibitor was evaluated by RT-qPCR, and the results are presented in Fig. 5a. Loss of PTPRG-AS1 inhibited proliferation (Fig. 5b) and induced apoptosis (Fig. 5c) in OVCAR3 and CAOV-3 cells, whereas cotransfection with miR-545-3p inhibitor abrogated the effects. Furthermore, si-PTPRG-AS1 clearly decreased the migratory (Fig. 5d) and invasive (Fig. 5e) abilities of OVCAR3 and CAOV-3 cells, which were restored by miR-545-3p inhibition.

**Fig. 5:** miR-545-3p silencing counteracts the si-PTPRG-AS1-induced inhibitory effects on EOC cells. **a** OVCAR3 and CAOV-3 cells were transfected with miR-545-3p inhibitor or NC inhibitor, and the miR-545-3p expression was measured by RT-qPCR. **b**, **c** The proliferation and apoptosis of OVCAR3 and CAOV-3 cells treated as described above were measured by CCK-8 assay and flow cytometry analysis, respectively. **e**, **e** The migratory and invasive abilities of the aforementioned cells were examined using Transwell cell migration and invasion assays. *P < 0.05 and **P < 0.01

The HDAC4 overexpression plasmid pc-HDAC4 induced HDAC4 protein expression in OVCAR3 and CAOV-3 cells (Fig. 6a) and was also used in the rescue experiments. The pc-HDAC4 or pcDNA3.1 plasmid in combination with si-PTPRG-AS1 was cotransfected into OVCAR3 and CAOV-3 cells, and functional experiments were performed. Upregulation of HDAC4 counteracted the effects of PTPRG-AS1 downregulation on the proliferation (Fig. 6b), apoptosis (Fig. 6c), migration (Fig. 6d), and invasion (Fig. 6e) of OVCAR3 and CAOV-3 cells. Cumulatively, these results indicated that PTPRG-AS1 promoted the oncogenicity in EOC cells by regulating the miR-545-3p/HDAC4 axis.

**Fig. 6:** HDAC4 reintroduction abolishes the inhibitory actions of PTPRG-AS1 knockdown on EOC cells. **a** The overexpression efficiency of pc-HDAC4 in OVCAR3 and CAOV-3 cells was determined by RT-qPCR. **b-e** si-PTPRG-AS1 in parallel with pc-HDAC4 or pcDNA3.1 was introduced into OVCAR3 and CAOV-3 cells. Proliferation, apoptosis, migration, and invasion were determined by CCK-8 assay, flow cytometry analysis, Transwell cell migration assay, and Transwell cell invasion assay, respectively. *P < 0.05 and **P < 0.01

### Knockdown of PTPRG-AS1 impairs EOC tumor growth in vivo

Using an in vivo tumor xenograft model, the effect of PTPRG-AS1 depletion on EOC tumor growth in vivo was explored. CAOV-3 cells transduced with lentivirus carrying sh-PTPRG-AS1 or sh-NC were subcutaneously injected into mice. The size of the subcutaneous tumors in the sh-PTPRG-AS1 group was smaller than that of those in the sh-NC group (Fig. 7a). Tumor growth (Fig. 7b) and weight (Fig. 7c) exhibited similar to that of tumor size. The subcutaneous tumors were excised, total RNA was isolated, and PTPRG-AS1 and miR-545-3p expression was measured. PTPRG-AS1 was downregulated (Fig. 7d) and miR-545-3p was upregulated (Fig. 7e) in the subcutaneous tumors originating from the sh-PTPRG-AS1 group. Furthermore, the HDAC4 protein level was lower in the sh-PTPRG-AS1 group than in the sh-NC group (Fig. 7f). Further IHC analysis also revealed that the tumor xenografts obtained from sh-PTPRG-AS1 group exhibited a decreased HDAC4 and Ki-67 expression (Fig. 7g). Consistent with our in vitro results, depletion of PTPRG-AS1 effectively impaired EOC tumor growth in vivo.

**Fig. 7:** The role of the PTPRG-AS1/miR-545-3p/HDAC4 pathway in EOC cell growth in vivo. **a** Representative images of subcutaneous tumors after injection with CAOV-3 cells transduced with lentivirus carrying sh-PTPRG-AS1 or sh-NC. **b** The growth curves of subcutaneous tumors after treatment with sh-PTPRG-AS1 or sh-NC. **c** The weight of subcutaneous tumors in sh-PTPRG-AS1 or sh-NC groups after treatment with sh-PTPRG-AS1 or sh-NC. **d**, **e** RT-qPCR measurement of the expression of PTPRG-AS1 and miR-545-3p in tumor xenografts. **f** The protein level of HDAC4 in tumor xenografts was determined by western blot analysis. **g** IHC analysis was applied to assess HDAC4 and Ki-67 expression in the tumor xenografts. **P < 0.01

## Discussion

With the development of gene sequencing, numerous lncRNAs have been identified that are dysregulated in the human genome [40]. A growing body of evidence has indicated that the dysregulated lncRNAs are closely related with the genesis and progression of EOC and are involved in the control of nearly all types of tumorigenic behavior [41–43]. However, a very small number of lncRNAs have been studied in EOC. Therefore, further elucidation of the detailed functions and relevant mechanisms of lncRNA in EOC is needed. In this study, we aimed to determine whether PTPRG-AS1 is implicated in the development of EOC.

PTPRG-AS1 is overexpressed in breast cancer [22], nasopharyngeal carcinoma [23], and gastric cancer [24]. Highly expressed PTPRG-AS1 is correlated with poor survival in patients with gastric cancer [24]. PTPRG-AS1 functions as a cancer-promoting lncRNA in nasopharyngeal carcinoma [23] and gastric cancer [24], and it is implicated in the regulation of several types of malignant processes. However, the expression and function of PTPRG-AS1 in EOC has not been defined. Our data revealed the overexpression of PTPRG-AS1 in EOC tissues and cell lines. High PTPRG-AS1 expression was indicative of poor prognosis in patients with EOC. Functionally, EOC cell proliferation, migration, and invasion in vitro and tumor growth in vivo were inhibited by the knockdown of PTPRG-AS1. In contrast, apoptosis was induced by PTPRG-AS1 depletion. These results highlight PTPRG-AS1 as a potential diagnostic and therapeutic target in EOC.

The specific function of lncRNAs are determined by their subcellular localization [44]. To illustrate how PTPRG-AS1 affects EOC progression, the localization of PTPRG-AS1 was predicted using two online bioinformatics tools, lncLocator and lncATLAS. PTPRG-AS1 was predicted to be mainly located in the cytoplasm, which was reconfirmed by subcellular fractionation studies. The observation suggested that PTPRG-AS1 regulates the oncogenicity of EOC cells by post-transcriptional regulation. In 2011, the ceRNA theory was proposed [45], which has been gradually recognized and accepted in the scientific community. In this theory, lncRNAs work as endogenous miRNA sponges, thereby protecting their target mRNAs from miRNA-mediated degradation [45].

Using a bioinformatics analysis, miR-545-3p was predicted to harbor a potential complementary binding site for PTPRG-AS1. RT-qPCR revealed that the silencing of PTPRG-AS1 resulted in a significant increase in miR-545-3p in EOC cells. Further studies indicated that miR-545-3p expression is weak in EOC and is inversely associated with PTPRG-AS1 expression. Luciferase reporter and RIP assays demonstrated that PTPRG-AS1 directly binds to miR-545-3p in EOC cells. In subsequent experiments, HDAC4 was determined to be the direct target of miR-545-3p. HDAC4 expression was decreased by miR-545-3p upregulation or PTPRG-AS1 depletion. Additionally, the PTPRG-AS1 deficiency-induced decrease in HDAC4 expression was abated following miR-545-3p inhibition. More importantly, RIP assay revealed that PTPRG-AS1, miR-545-3p, and HDAC4 were present in the same RISC. The collective results validate PTPRG-AS1 as a molecular sponge that sequesters miR-545-3p and consequently increases HDAC4 expression in EOC cells.

Differentially expressed miR-545-3p has been observed in diverse human malignancies [46–48]. In EOC, miR-545-3p is downregulated in EOC tissues and cell lines [34]. Patients with EOC characterized by low miR-545-3p expression have a shorter overall survival than those with high miR-545-3p expression [34]. Consistent with this result, the decrease of miR-545-3p expression in EOC was verified in our study and its upregulation suppressed cell growth and metastasis by directly targeting HDAC4. HDAC, a member of the histone deacetylase family, is overexpressed in EOC and is associated with poor overall and progression-free survival in patients with EOC [49]. HDAC4 exerts a pro-oncogenic function during EOC progression and participates in the control of a wide range of tumorigenic behaviors [37–39]. In this study, our results confirmed the control of HDAC4 expression in EOC cells by PTPRG-AS1/miR-545-3p axis. Furthermore, rescue experiments demonstrated that PTPRG-AS1 knockdown-mediated anti-oncogenic activities in EOC cells were reversed by increasing the output of the miR-545-3p/HDAC4 axis. Altogether, PTPRG-AS1, miR-545-3p, and HDAC4 form a ceRNA regulatory network that promotes the malignant characteristics of EOC cells. These results may provide new insights into the role of the lncRNA/miRNA/mRNA pathway in the initiation and progression of EOC.

Our study provided sufficient evidence that PTPRG-AS1 acts as an oncogenic lncRNA to aggravate the malignancy of EOC through the miR-545-3p/HDAC4 ceRNA network. The PTPRG-AS1/miR-545-3p/HDAC4 pathway may lead to novel strategies for the prevention, diagnosis, and treatment of EOC.

## Data Availability

The analyzed data sets generated during the study are available from the corresponding author on reasonable request.

## Abbreviations

EOC: Epithelial ovarian cancer
FBS: Fetal bovine serum
HIF: Hypoxia-Inducible Factor
NC: Negative control
PBS: Phosphate buffer saline
RISC: RNA-induced silencing complex
WT: Wild-type
lncRNA: long non-coding RNA
PTPRG-AS1: RNA PTPRG antisense RNA 1
miRNA: microRNA
